# Weipiling ameliorates gastric precancerous lesions in Atp4a^−/−^ mice

This article has been retracted.

**DOI:** 10.1186/s12906-019-2718-y

**Published:** 2019-11-19

**Authors:** Wei Liu, Zi-ming Zhao, Yuan-liang Liu, Hua-feng Pan, Li-zhu Lin

**Affiliations:** 1 Guangzhou University of Chinese Medicine, Guangzhou, 510405 Guangdong China; 2 Integrative Cancer Centre, the First Affiliated Hospital of Guangzhou, University of Chinese Medicine, Guangzhou, China; 3 Guangdong Province Engineering Technology Research Institute of T.C.M, Guangzhou, 510095 China

**Keywords:** Gastric precancerous lesions, Traditional Chinese medicine, Atp4a^−/−^mice, Weipiling, Glycolysis, mTOR/HIF-1α pathways

## Abstract

**Background:**

Altered cellular metabolism is considered to be one of the hallmarks of cancer (Coller, Am J Pathol 184:4–17, 2014; Kim and Bae, Curr Opin Hematol 25:52–59, 2018). However, few studies have investigated the role of metabolism in the development of gastric precancerous lesions (GPLs). Weipiling (WPL), a traditional Chinese medicine formula for treatment of GPLs. In this study, we evaluated the amelioration of GPLs by WPL and investigated the possible role of WPL in regulating glucose metabolism.

**Methods:**

Firstly, the major components of WPL are chemically characterized by HPLC analytical method. In this study, we chose the Atp4a^−/−^ mouse model (Spicer etal., J Biol Chem 275:21555–21565, 2000) for GPL analysis. Different doses of WPL were administered orally to mice for 10 weeks. Next, the pathological changes of gastric mucosa were assessed by the H&E staining and AB-PAS staining. In addition, TUNEL staining was used to evaluate apoptosis, and we further used immunohistochemically labelled CDX2, MUC2, ki-67, PTEN, and p53 proteins to assess the characteristic changes of gastric mucosa in precancerous lesions. The levels of such transporters as HK-II, PKM2, ENO1, MPC1, and LDHA were determined by Western blot analysis. Finally, we assessed the expression of mTOR, HIF-1α, AMPK, Rheb, TSC1 and TSC2 protein in the gastric mucosa of Atp4a^−/−^mice.

**Results:**

In this work, we evaluated the protective effect of WPL on gastric mucosa in mice with precancerous lesions. The aberrant apoptosis in gastric mucosa of gastric pre-cancerous lesions was controlled by WPL (*P<0.05*). Furthermore, WPL suppressed the expression of CDX2, MUC2, ki-67, PTEN and p53, as the levels of these proteins decreased significantly compared with the model group (*P*<*0.05*). In parallel, WPL significantly suppressed the expression of transporters, such as HK-II, PKM2, ENO1, MPC1 and LDHA (*P<0.05*). In addition, mTOR, HIF-1a, AMPK, Rheb, TSC1 and TSC2 protein levels in gastric mucosa of Atp4a^−/−^ mice in the high- and low-dose WPL groups were significantly lower than those in the model group (*P<0.05*), while the expression of TSC1 and TSC2 protein was significantly higher (*P<0.05*).

**Conclusions:**

Conclusively, WPL could ameliorate GPLs in Atp4a^−/−^ mice by inhibiting the expression of transporters and suppressing the aberrant activation of mTOR/HIF-1α.

## Background

Gastric cancer (GC) is the fifth most frequently diagnosed cancer and the third most common cause of cancer-related mortality worldwide [1]. Therefore, the treatment of precancerous lesions with malignant transformation potential is of great significance to reduce the incidence of GC. Chronic inflammation of the gastric mucosa leads to atrophic changes and damage to glandular cells, which are replaced by intestinal-type epithelium. GPLs are a kind of GC that are closely related to the pathological changes of gastric mucosa during the development of gastric cancer [2]. Gastric atrophy and IM are classified as precancerous lesions [3]. Previous studies have identified a direct link between GC and a high prevalence of GPLs worldwide [4–6]^.^ Thus, blocking gastric precancerous cells from malignant transformation is crucial for early detection and prevention of GC.

Generally, GPLs require endoscopic resection due to the potential for progression to carcinoma. However, repeated endoscopic examination with biopsies may impose a physical, psychological, and financial burden on the patient [7]. Therefore, different strategies, such as preventive or alternative medicine, merit further investigation. Chinese medicine owing to its nature, vast resources, and low cost, has been used as medicine for thousands of years is used in the treatment of gastrointestinal diseases in a variety of ways. Therefore, the study of Chinese medicine in the treatment of GPLs needs further investigation, this study provides preliminary insights into its mode of action as an anti-GPL agent.

The Warburg effect in tumour cells involves the uptake of high levels of glucose, enhanced glycolysis, and the metabolism of pyruvate to lactic acid, rather than oxidative phosphorylation, to generate energy under aerobic conditions. This effect is closely related to the occurrence, invasion, metastasis, drug resistance, and poor prognosis of GC [8]. As such, dysfunctional changes in cellular energy metabolism in GPLs warrant further investigation.

Replication of disease models is an effective tool for studying disease pathogenesis and treatment. For the study of GPL, researchers used chemical drug induction and *HP* infection methods, but there are limitations in model replication time, large individual differences, and unstable models, thus affecting the study of GPL. As we reported before, with the development of genetic engineering technology, knockout mice are gradually being used to study precancerous lesions [9]. The phenotypic progression to IM observed in the Atp4a^−/−^ mouse model is similar to the evolution of gastric cancer in humans [9–11], as initially described by Correa [12].So in this research, we choose the Atp4a^−/−^ mice to simulate GPL.

Weipiling (WPL) is based on an improved version of Sijunzi decoction. Weipixiao, another Chinese medicine formula, also based on the Sijunzi decoction, has shown a certain protective effect on precancerous lesions [13].Weipiling can be prepared from conventional decoction of eight Chinese medicinal herbs including *Hedysarum multijugum* Maxim(Huang-qi), *Pseudostellaria heterophylla* (Miq.) Pax (Tai-zi-shen),*Atractylodes macrocephala* Koidz (Bai-zhu), *Poria cocos* (Schw) Wolf (Poria) (Fu-ling), *Panax notoginseng* (Burk.) F. H. Chen (*P. notoginseng) (*San-qi*)*, *Curcuma zedoaria* (Christm.), Roscoe (E- zhu), *Hedyotis diffusa* Willd (She- she-cao) and *Hericium erinaceus* (Rull ex F.) Pers (Hou-gu-jun). These Chinese medicinal materials described above have pharmacological effects of replenishing qi to invigorate the spleen, and removing blood stasis and detoxify, however, the Weipixiao is only the “Yi Qi Hua Yu” decoction. Experimentally, some WPL individuals exhibited potential anticarcinogenesis activities. *Astragalus membranaceus* induced by apoptosis of human gastric carcinoma via intrinsic mitochondrial pathways [14], Clinical research showed that *Atractylodes macrocephala* Koidz can be beneficial for treating cancer cachexia [15], *Poria cocos* (Schw.) Wolf (Poria) arrest Cell-cycle and induce apoptosis of breast carcinoma [16]. *Curcuma zedoaria* inhibited AGS human gastric cancer cell viability by activating caspase-8, caspase-9, caspase-3, and PARP, which contributed to apoptotic cell death in AGS human gastric cancer cells [17]. *Hedyotis Diffusa* Willd. has been using to treat malignant tumors, and showed significant effective on malignant tumors of gastric, colon, rectal [18, 19]. The specific mechanism governing this effect is unknown, thus, this study aimed to assess WPL efficacy in the GPL mice and explore its potential mechanisms.

## Methods

### Preparation of WPL

The components of the WPL formulation are shown in Table 1. These formulations were purchased from the First Affiliated Hospital of Guangzhou University of Chinese Medicine. The multi-herbs were boiled with distilled water, refluxed, and concentrated into a mixture containing 0.2 g/mL crude drugs. Vitacoenzyme tablets (VIT) were supplied by Guangxi Dahai Sunshine Pharmaceutical Co. (No.160202).

**Table 1:** Components of the WPL formulation

Chinese herbal name in Pinyin name	Species name	Amount (g)
Huang-qi	*Hedysarum multijugum* Maxim	20
Tai-zi -shen	*Pseudostellaria heterophylla* (Miq.) Pax	15
Bai-zhu	*Atractylodes macrocephala* Koidz	10
Fu- ling	*Poria cocos* (Schw) Wolf (Poria)	12
San- qi	*Panax notoginseng* (Burk.) F. H. Chen (*P. notoginseng)*	3
E- zhu	*Curcuma zedoaria* (Christm.), Roscoe	10
She-she-cao	*Hedyotis diffusa* Willd	15
Hou-gu-jun	*Hericium erinaceus* (Rull ex F.) Pers	15

### Animals and drug administration

All of the experiments involving animals were in accordance with the guidelines of the Institutional Animal Care and Use Committee of Guangzhou University of Chinese Medicine (Guangzhou, China). In addition, all of the procedures were approved by the Animal Care Ethics Committee of Guangzhou University of Chinese Medicine (No. S2017089). All efforts were made to minimize the suffering of animals as much as possible. Sixty 6-week-old male Atp4a^−/−^ C57Bl/6 mice (specific pathogen-free) were obtained from Shanghai Model Organisms Centre Inc. Mice were maintained on standard laboratory conditions with food and water ad libitum for the duration of the study. The mice were randomly divided into control, model, VIT, and WPL groups according to various interventions: animals in the VIT group were administered 0.2 g/kg/d vitacoenzyme, and animals in the high-dose WPL group and low-dose WPL group were given 15 g/kg/d and 7.5 g/kg/d WPL, respectively. All mice, except for the control mice, underwent hunger-satiety shift every other day. At the beginning of the 10th week, the treated mice were administered WPL or VIT by gastrogavage for 10 consecutive weeks, while the control and the model mice were treated similarly with corresponding volume of distilled water once daily. At the end of the 10th week, all the experimental mice were humanely terminated with sodium pentobarbital (60 mg/kg, injected intraperitoneally) diluted with phosphate-buffered saline (PBS). Each treatment was placed in a 1 ml syringe as dictated by the volume of injectate. A new 25 G 5/8″ hypodermic needle was attached to each syringe for injection. Two-person injection technique used in the study, with one person holding the mice in dorsal recumbency (head down) and the second person gently restraining the right pelvic limb to facilitate intraperitoneal injection in to the right caudal quadrant. The left thoracic wall was then auscultated continuously with a stethoscope to identify cessation of heartbeat (CHB). Following CHB, each animal was carefully removed from the chamber and positioned in dorsal recumbency for necropsy examination.

### HPLC-MS analysis of WPL decoction

To confirm the stability of the decoction within the experimental period, HPLC-MS (Thermo Fisher, Thermo Scientific triple stage quadrupole) was employed to determine the contents of the eight major constituents of the WPL decoction. Isoflavone glucoside and notoginsenoside R1 were used as standard substances. Ultra-pure water was obtained from a Milli Q-plus system (Millipore, France). Briefly, WPL powder (0.25 g) was dissolved in 25 mL of a methanol solution in an ultrasonic bath for 30 min. The solution was filtered through a 0.22-μm membrane filter. An ESI ion source was used for the MS/MS analysis. The Vaporizer Temperature was 350 °C, Spray Voltage 3000 v, Sheath Gas Pressure was 30, Aus Gas Pressure was 10 v, Lon Sweep Gas Pressure was 0v, and Caoillary Temperature was 300 °C. All the data were analysed by Chemstation software.

### Pathological examination

For histology, the gastric tissue sections were excised and fixed in 10% buffered formalin, pH 7.4. Samples were dehydrated by being passed through a series of alcohols with incremental concentrations, equilibrated in xylene for 10–15 min and embedded in paraffin; the paraffin blocks were cut into approximately 3-μm sections using a microtome. The prepared specimens were stained with haematoxylin and eosin (H&E) (Beyotime, C0105, China) or alcian blue-periodic acid-Schiff (AB-PAS) (BASO, 615041, China). The staining steps were carried out according to the kit instructions.

### Western blot analysis

Thirty micrograms of protein were separated via sodium dodecyl sulfate polyacrylamide gel electrophoresis and transferred to nitrocellulose membranes. Immunolabelling was performed using rabbit mTOR (1:1000 dilution; Abcam: ab109268, USA), HIF-1a (1:500 dilution; Millipore: MAB5382, USA), AMPK (1:1000 dilution; CST: 2535, USA), Rheb (1:1000 dilution; CST: 13879, USA), TSC1 (1:1000 dilution; CST:6935, USA), TSC2 (1:1000 dilution; CST: 3990, USA), MPC1 (1:1000 dilution; CST: 14462, USA) and β-actin (1:1000 dilution; CST: 4967, USA) antibodies. Then, the membranes were incubated with HRP-linked anti-rabbit IgG (1 mg/mL, dilution; Millipore: AP132P, USA) for 1 h. The protein bands were detected using an ECL reagent kit (GE Healthcare). Optical density was normalized against β-actin.

### TUNEL assay

TUNEL staining was performed using an In-Situ Cell Death Detection Kit (No. 11684795910; Roche, Stockholm, Sweden) according to the manufacturer’s instructions. Nuclei were stained with 4′,6-diamidino-2-phenylindole (DAPI; Solarbio, Beijing, China).

### Immunohistochemistry assay

The paraformaldehyde-fixed gastric tissues were embedded in paraffin and cut into sections, dewaxed and hydrated. After blocking the appropriate antisera, the sections were incubated with CDX2 (1:100 dilution; Abcam, ab157524), MUC2 (1:100 dilution; Abcam, ab76774), ki-67 (1:100 dilution; Abcam, ab16667), p53 (1:100 dilution; Millipore, #CBL404), and PTEN (1:100 dilution; Abcam, ab238032). Then, the sections were incubated with anti-rabbit or anti-mouse IgG (Boshide Biological Technology, Wuhan, China). Positive signals were visualized using a diaminobenzidine kit (GTVisionTM III Detection System/Mo&Rb; Gene Group Holdings, Shanghai, China), and the sections were counterstained with haematoxylin. Image-Pro was used to analyse the integrated optical density (IOD) and area of each picture. The mean density (IOD/area) was used to analyse the protein expression.

### Statistical analysis

All experimental values are expressed as mean values ± SD. GraphPad Prism 5.0 software was used to analyse the data. One-way analysis of variance (ANOVA) was used to analyze statistical differences between groups or Student’s *t*-test was performed as appropriate. *P* < 0.05 was considered to be significant.

## Results

### HPLC profile

WPL possesses an excellent inhibitory ability against GPLs, as revealed by our previous clinical trials and animal testing; therefore, we investigated the major constituents of WPL multi-herbal mixtures. Figure 1 shows the HPLC chromatograms of WPL reference samples (A, C) and test samples (B, D). The retention times of the major chemical constituents were 0.81 min (isoflavone glucoside) and 0.71 min (notoginsenoside R1).

**Fig. 1:** HPLC chromatogram of WPL text samples (**b, d**) and reference samples (**a, c**). Note: Peak 1 is isoflavone glucoside, and Peak 2 is notoginsenoside R1

### WPL inhibited the progression of gastric precancerous lesions

For the GPL animal model, Atp4a^−/−^ mice were used to establish the GPL mouse model by multiple factors, and the procedure lasted 10 weeks. To investigate the anti-GPL effect of WPL, we examined gastric epithelial dysplasia lesions in H&E-stained sections of gastric tissues. Compared with the control group, the gastric mucosa in the model group was pale and exhibited poor elasticity, little mucus, fine wrinkles, increased nuclear-cytoplasmic ratio, loss of nuclear polarity and occasional binucleation. Inflammatory infiltration was variable and sometimes extensive. Some submucosal vascular hyperplasia, erosion or granular changes were observed (Fig. 2a).

**Fig. 2:** Histological evaluation of gastric epithelial dysplasia and intestinal metaplasia (H&E staining, 400×). **a** The model gastric epithelium displayed dysplasia pathology characterized by glandular architectural abnormalities. After WPL intervention, these dysplasia pathological alterations, especially irregularities of glandular structure, were regressed to varying degrees. *n* = 6 in each group. **b** Histological evaluation of gastric intestinal metaplasia (AB-PAS staining, 200×). Neutral mucins present in normal mucosa were stained red. Sialomucins expressed only in intestinal-type metaplasia (IM) were stained blue. Images of the model gastric epithelium depicted prominent IM lesions, which were dramatically reduced after WPL administration. *n* = 5 in each group

In most WPL-treated Atp4a^−/−^ mice, the decoction shows a strong effect in model animal growth and inhibited atypical hyperplasia and inflammatory infiltration in the Atp4a^−/−^ mice; in contrast, this GPL-rescuing effect was not observed in most VIT-treated mice. These observations suggest that WPL can inhibit and even reverse the dysplastic process (Fig. 2a), which appears to explain the effect of WPL in the clinic.

We evaluated the degree of IM lesions in gastric tissues by AB-PAS staining. As depicted in Fig. 2b, neutral mucins present in normal mucosa were stained red, and gastric specimens from controls did not exhibit IM lesions. In model mice, sialomucins expressed only in IM lesions were stained blue, indicating that IM lesions were widespread. In treated mice, IM lesions regressed slightly in VIT-treated mice. In comparison, IM lesions were regressed visibly in WPL-treated mice. Our observation revealed that WPL has a potent anti-IM-lesion capacity in GPL mice (Fig. 2b).

### WPL reduced the CDX2, MUC2, Ki-67, p53 and PTEN levels in GPL tissues

To investigate the features of the acute gastric mucosal lesion in Atp4a^−/−^ mice, we applied immunohistochemistry to examine the CDX2, MUC2, Ki-67, PTEN and p53 levels in Atp4a^−/−^ mice gastric tissues and determined whether WPL possessed an inhibitory effect on intestinal metaplasia and malignant proliferation of gastric mucosa.

Caudal-related homeobox transcription factor 2 (CDX2) is an intestinal-specific transcription factor that has been strongly implicated in the development of intestinal epithelial cells, where it regulates intestinal markers, including mucin 2 (MUC2). Positive CDX2 and MUC2 staining were increased in model mouse gastric tissues compared with normal gastric mucosa (Fig. 3). Moreover, we found that WPL could visually reduce the number of CDX2- and MUC2-positive cells in the majority of GPL tissues, as shown in Fig. 3. Through semiquantitative analysis, elevated CDX2 and MUC2 protein expression levels were observed in GPL mucosa compared to normal mucosa (*P* < 0.01). After WPL intervention, we found a clear downtrend, though without statistical significance of CDX2 and MUC2 levels in gastric mucosa (*P* < 0.01). Our results indicated that WPL treatment may produce regulatory effects on the IM of gastric mucosa, which further verifies the AB-PAS staining result in Fig. 2b. Mucins are the major components of gastric mucus which protects gastric mucosa against bacterial infection, proteolytic enzymes and hydrochloric acid.

**Fig. 3:** Evaluation of CDX2 and MUC2 in gastric mucosa. **a** Representative immunohistochemical staining of CDX2 in the mouse gastric mucosa. **b** Analysis of gastric mucosa total protein of CDX2. **c** Representative immunohistochemical staining of MUC2 in the mouse gastric mucosa. **d** Analysis of gastric mucosa total protein of MUC2. Data are expressed as the mean ± SD. ** indicates *P* < 0.01 compared with the control group. ^*#*^ indicates *P* < 0.05 and ^##^ indicates *P* < 0.01 compared with the model group (IHC, 400×). *n* = 5 in each group

The cell proliferation nuclear antigen Ki-67 is a gene related to the cell cycle, which is indispensable in cell proliferation. Therefore, the protein of Ki-67 in the gastric mucosa was documented (Fig. 4). The gastric mucosa expression of Ki-67 in the model group was increased compared to the control group (*P* < 0.01). The upregulated Ki-67 expression was decreased by VIT and WPL treatment (*P* < 0.01), suggesting that WPL significantly inhibits the malignant proliferation of gastric mucous membrane cells. Thus, WPL could effectively inhibit dysplasia of gastric mucosa in GPL mice as shown in Fig. 2a.

**Fig. 4:** Evaluation of ki-67 in gastric mucosa. **a** Representative immunohistochemical staining of ki-67 in the mouse gastric mucosa. **b** Analysis of gastric mucosa total protein. Data are expressed as the mean ± SD. ** indicates *P* < 0.01 compared with the control group. ^##^ indicates *P* < 0.01 compared with the model group (IHC, 400×). *n* = 5 in each group

Both PTEN (phosphatase and tensin homolog) and p53 are known as cancer suppressor genes, and mutations of these genes occur frequently in various types of carcinoma. Therefore, in this study, we investigated both p53 and PTEN in gastric mucosa. As shown in Fig. 5, immunohistochemistry assays confirmed that the expression of p53 in the model group was increased compared with the control group (*P* < 0.01), and WPL treatment reduced the expression of p53 (*P* < 0.01). Furthermore, the expression of PTEN was lowered in the model group (*P* < 0.01), and a high dose of WPL treatment improved the level of PTEN in the gastric mucosa (*P* < 0.01). Taken together, these results suggested that WPL regulates the mutation of the oncogene.

**Fig. 5:** Evaluation of p53 and PTEN in gastric mucosa. **a** Representative immunohistochemical staining of p53 in the mouse gastric mucosa. **b** Analysis of gastric mucosa total protein of p53. **c** Representative immunohistochemical staining of PTEN in the mouse gastric mucosa. **d** Analysis of gastric mucosa total protein of PTEN. Data are expressed as the mean ± SD. ** indicates *P* < 0.01 compared with the control group. ^##^ indicates *P* < 0.01 compared with the model group (IHC, 400×). *n* = 5 in each group

### Effects of WPL on apoptosis

TUNEL staining was used to determine the role of apoptosis in gastric injuries in mice with GPLs. The number of TUNEL-positive cells was significantly decreased in the model group (*P* < 0.01) (Fig. 6). WPL increased the clumps of condensed heterochromatin, which is consistent with the observation of VIT (*P* < 0.05). These results suggested that apoptosis might be responsible for gastric dysfunction in GPLs and WPL similar to VIT promoted the cellular apoptosis of the stomach from GPL model mice.

**Fig. 6:** Effects of WPL on apoptosis. **a** The images of TUNEL positive cells were captured by a fluorescence microscope (× 200). left panel: DAPI staining; middle panel: TUNEL assay, right panel: merged image showing the results of DAPI staining and the TUNEL assay. **b** Quantitative result of TUNEL assay was analyzed. Data are expressed as the mean ± SD. ** indicates *P* < 0.01 compared with the control group. indicates *P* < 0.05 and indicates *P* < 0.01 compared with the model group. n = 5 in each group

### WPL influences the mTOR/HIF-1a signalling pathway to regulate aerobic glycolysis

The mTOR/HIF-1a pathway has been reported in the literature to regulate aerobic glycolysis and promote cancer cell apoptosis and proliferation, resulting in cancer development. As cancer cells activate aerobic glycolysis, glucose is metabolized to lactate. The lactate synthesized in the cytosol is then secreted outside the cells by monocarboxylate transporters, producing and maintaining the acidic microenvironment. The lower extracellular pH microenvironment could also accelerate malignant biological behaviours, including invasion, metastasis, and cellular proliferation. To ascertain the mechanism by which the WPL decoction ameliorated GPLs in Atp4a^−/−^ mice, we analysed the expression levels of HK-II, PKM2, ENO1, MPC1 and LDHA protein in decoction-fed Atp4a^−/−^ mouse gastric mucosa by Western blotting (Fig. 7). Compared with the non-fed group, the WPL-fed group exhibited decreased HK-II, PKM2, ENO1 and LDHA levels in tissue and upregulated MPC1 levels (*P* < 0.01). We further examined the effects of WPL on the mTOR/HIF-1a pathway. Compared with the control group (Figs. 8 and 9), the WPL can lower the protein of mTOR, HIF-1a, AMPK, Rheb, TSC1 and TSC2 (*P* < 0.01). These results suggested that WPL might inhibit aerobic glycolysis of gastric mucosal cells in pre-cancerous lesions through the mTOR/HIF-1a signalling pathway.

**Fig. 7:** Expression of key enzymes for glucose metabolism in gastric tissue treated with WPL (**a-e**) Western blotting was used for the analysis. (**f**) Expression of proteins in the mouse gastric. Data are expressed as the mean ± SD. * indicates *P* < 0.05 and ** indicates *P* < 0.01 compared with the control group. ^*#*^ indicates *P* < 0.05 and ^##^ indicates *P* < 0.01 compared with the model group. *n* = 5 in each group

**Fig. 8:** Expression of mTOR and HIF-1α protein. **a-b** Western blotting was used for the analysis. **c** Expression of proteins in the mouse gastric. Data are expressed as the mean ± SD. ** indicates *P* < 0.01 compared with the control group. ^##^ indicates *P* < 0.01 compared with the model group. *n* = 5 in each group

**Fig. 9:** Effect of WPL on AMPK pathway protein levels in gastric epithelial cells. **a-d** Western blotting was used for the analysis. **e** Expression of proteins in the mouse gastric. Data are expressed as the mean ± SD. * indicates *P* < 0.05, and** indicates *P* < 0.01, compared with the control group. ^##^ indicates *P* < 0.01 compared with the model group. *n* = 5 in each group

The cancerization of gastric mucosa epithelial cell is a gradual process. The results of HE and AB-PAS staining suggest that the gastric mucosa of Atp4a^−/−^ mice display the intestinal metaplasia and the adenomatous dysplasia with a back -to -back gland pattern. To study the biological features, we used CDX2, MUC2 for cell differentiation, p53 for cell cycle control, Ki-67 for proliferation. Immunohistochemical staining for CDX2, MUC2, Ki-67, P53 and PTEN was performed, and their expression levels were evaluated in the mucosa. The results, including western blot analysis, showed the characteristics of intestinal metaplasia, dysplasia and abnormal energy metabolism of gastric mucosa in mice with GPL.

## Discussion

The essential difference between cancer cells and normal cells is the aberrant proliferative capacity of cancer cells, as cancer cells have an excessive need for nutrients and energy [20]. Aerobic glycolysis was observed in GC tumour tissue, but few scholars have studied the metabolic patterns of poplar in GPLs, which was investigated in this study. The development of GC is a multi-factor, multi-step, progressive pathological process [21]. It is highly important to study the mechanism of GPLs to clarify the mechanism of gastric carcinogenesis. Our results show that WPL decreased the expression of key enzymes in aerobic glycolysis and gastric mucosa injury in the Atp4a^−/−^ mice, suggesting that it ameliorates gastric mucosa of GPLs via regulating the mTOR/HIF-1α signal channel.

In this project, all Atp4a^−/−^ mice exhibited GPLs, which ranged from IM to Dys. After WPL administration, IM lesions were markedly regressed in most cases of Atp4a^−/−^ mice. We also found that WPL could arrest and even reverse the majority of mild and moderate dysplasia. WPL decreased the formation of clumps of condensed heterochromatin, which is consistent with the observation of VIT. Our observations reinforce the view that GPLs can be blocked and reversed.

The homeostasis of gastric mucosal epithelial cells is maintained by the balance between apoptosis of damaged or senescent cells and the proliferation of normal gastric epithelial cells [22]. Impairment of apoptosis was observed in GPL and gastric cancer [23, 24]. Therefore, dysregulation of apoptosis might be one of the main causes of gastric cancer development. In our study, we found that WPL treatment decreased GPL incidence and enhanced gastric epithelial apoptosis.

Most gastric cancers develop via an IM-Dys-carcinogenic pathway [25]. Therefore, to study the clinically effective mechanism of WPL in GPLs, we studied the biological characteristics of gastric mucosa before and after treatment. Notably, in this study, we found that WPL could reduce the expression of CDX2 and MUC2, supporting the hypothesis that the staining of AB-PAS could be reversed by WPL. To the best of our knowledge, this study is the first to investigate GPLs and their relationship to Ki-67 protein expression. Ki-67, a nuclear antigen, is expressed in all phases of the cell cycle, except G0 [26], and can therefore be used as a cell proliferation marker. In our study, we found that normal gastric epithelial cells showed a low proliferative index and that the gastric tissue of GPLs showed a high proliferative index. With comprehensive research on the molecular biology of cancer, it has been found that there are close associations among p53, PTEN, the mTOR/HIF-1α signalling pathway and growth, proliferation, infiltration, expansion, and metastasis of malignant cells [27]. In gastric lesions, an increasing frequency of p53 mutations is observed in *H. pylori* infection, a key player in gastric carcinogenesis, intestinal metaplasia, gastric dysplasia and gastric carcinoma [28]. Currently, p53 is also involved in energy reprogramming of malignant tumours, maintaining the balance between tumour cell aerobic metabolism and AEG by regulating glucose metabolism [29]. PTEN is a tumour suppressor gene, and mutations in PTEN are associated with a large number of tumours; only p53 mutations are associated with more tumours. In our study, the protein expression of PTEN in GPL tissues was significantly decreased compared with the control group, and in contrast, the protein expression of p53 in the model group was significantly increased compared with that in normal tissues. Interestingly, a previous study indicated that PTEN in oesophageal cancer tissues presented a significantly lower expression compared with those in adjacent normal tissues [30]. More importantly, WPL could suppress the anti-oncogene accumulation of p53 and PTEN activation. This result supports the hypothesis that energy metabolic recombination inhibition plays a beneficial role in WPL-treated GPLs.

The metabolic changes dominated by the Warburg effect have recently been referred to as metabolic reprogramming, and studies of these changes have provided a deeper understanding of tumour cell metabolism. Key enzymes in glycolysis primarily involve changes in metabolic reprogramming. Moreover, interventions targeting these molecules have been found to affect not only the metabolic profile of GC cells but also the genesis, proliferation, invasion, and metastasis of GC cells [31]. However, the role of cell metabolism in GPLs is less clear. In this study, as expected, upregulated protein expression of HK-II, PKM2, ENO1 and LDHA and downregulated protein expression of MPC1 were observed in gastric mucosa from Atp4a^−/−^ mice compared tonormal mucosa. Our results demonstrate that the metabolic reprogramming observed in GPLs is partly driven by aberrant activation of metabolic-related enzymes, suggesting their involvement in malignant transformation. We also investigated whether inhibition of key enzymes is involved in the underlying mechanisms of WPL-mediated attenuation of metabolic reprogramming. Interestingly, after WPL intervention, a decrease in metabolic-related enzyme levels was frequently concurrent with the inhibition of the mTOR/HIF-1α pathway. Hence, this expression of enzymes regulated by the mTOR/HIF-1α pathway mitigating effect might contribute to the metabolic reprogramming activity of WPL against precursor lesions. Additionally, WPL can restrict cellular differentiation by negatively regulating AMPK-mediated signalling.

In recent years, more scientific researchers have done in-depth research on the treatment of GPL. However, they used the rats treated with MNNG to demonstrate GPL [24, 32, 33]. this method has the limitation that the pathologic degree of the time-consuming and non-uniform digress of pathological degree of the model. In this article, the Atp4a^−/−^ mice was used to established GPL, the gastric mucosa of 10-week old mice showed the intestinal metaplasia, dysplasia, which is more closely rated to the clinical patients of the premalignant lesions of the clinical gastric cancer. The limitations of this study are that the vitro cell model of GPL is not established until now, so we elaborate the effect of gastric mucosa protection of WPL may through regulating glucose metabolism in GPL mice.

Our HPLC analysis revealed that isoflavone glucoside and notoginsenoside R1 might be the potential anti-metabolic reprogramming candidates of WPL. Isoflavone glucoside is extracted from *Astragalus membranaceus*, which displayed a protective action against inflammation and gastrointestinal cancers [34]. Ginsenoside Rg1 has been reported to attenuate chronic atrophic gastritis in rats [35]. In addition, ginsenoside Rb1 potentiated the improvement of energy metabolism, and the underlying mechanism might be associated with promoting the activation of AMPKα1/2, thereby enhancing the expression of GLUT3 [36]. In the present study, WPL could adjust the mTOR/HIF-1α pathway to protect against metabolic reprogramming.

## Conclusions

In conclusion, by examining Atp4a^−/−^ mice, our research provides direct evidence that WPL downregulates the mTOR/HIF-1α pathway to suppress energy metabolism reprogramming in mice with GPLs. This approach may provide a theoretical basis for the clinical treatment of GPLs.

## Data Availability

The datasets used and analyzed during the current study available from the corresponding author on reasonable request. All data generated or analysed during this study are included in the manuscript.

## Abbreviations

CDX2: Caudal-related homeobox transcription factor 2
CST: Cell Signaling Technology
GC: Gastric cancer
IM: Intestinal metaplasia
VIT: Vitacoenzyme tablets
WPL: Weipiling
